The article "Adoption of Wireless Network and Artificial Intelligence Algorithm in Chinese-English Tense Translation" was published in 2022. Journal: Comput Intell Neurosci.

# Adoption of Wireless Network and Artificial Intelligence Algorithm in Chinese-English Tense Translation

**DOI:** 10.1155/2022/1662311

**Published:** 2022-06-11

**Authors:** Xiaojing Li

**Affiliations:** Foreign Language Department, Henan University of Chinese Medicine, Zhengzhou 450000, Henan, China

## Abstract

In order to solve the problem of tense consistency in Chinese-English neural machine translation (NMT) system, a Chinese verb tense annotation model is proposed. Firstly, a neural network is used to build a Chinese tense annotation model. During the translation process, the source tense is passed to the target side through the alignment matrix of the traditional Attention mechanism. The probability of the candidate words inconsistent with the corresponding tense of source words in the candidate translation word set is also reduced. Then, the Chinese-English temporal annotation algorithm is integrated into the MT model, so as to build a Chinese-English translation system with temporal processing function. The essence of the system is that, in the process of translation, Chinese-English temporal annotation algorithm is used to obtain temporal information from Chinese sentences and transfer it to the corresponding English sentences, so as to realize the temporal processing of English sentences and obtain the English sentences corresponding to the tenses of the original Chinese sentences. The experimental results show that the Chinese tense annotation model of bidirectional long short-term memory (LSTM) is more accurate for the prediction of Chinese verb tense, so the improvement effect of NMT model is also the most obvious, especially on the NIST06 test set, where the BLEU value is increased by 1.07%. As the mainstream translation model, the transformer model contains multihead Attention mechanism, which can pay attention to some temporal information and has a certain processing ability for temporal translation. It solves the tense problems encountered in the process of MT and improves the credibility of Chinese-English machine translation (MT).

## 1. Introduction

In the 21st century, with the advent of the era of knowledge economy, information processing has become particularly important. As the main carrier of information, language is very important in the application of natural language processing technology in information processing, including automatic translation between natural languages represented by machine translation (MT) [1, 2]. Since the successful development of the first electronic computer, some scholars have begun to study MT. With the rapid development of computer technology and modern linguistics, new progress has been made in MT, and many commercial and practical MT systems have emerged [3]. Information technology represented by the Internet is in a period of rapid development, and MT technology is entering an unprecedented period of opportunity driven by social and economic benefits. Chinese and English are the two most populous languages in the world, and language collisions are very frequent. Automatic translation between Chinese and English is conducive to accelerating the process of China's modernization and has attracted extensive attention [4, 5].

MT is the process of translating one natural language into another through computer. The concept of MT appeared after the birth of the first computer. People began to use machines to realize automatic translation between two languages, which liberated a lot of artificial mental labor [6]. The processing of natural language is divided into two camps: empiricism and rationalism. Rationalism is a common method in the temporal processing of Chinese-English MT. Roy and Ghosh [7] researched some additional information that humans took into account in the translating process of tense and tried to determine where to focus in the automatic extraction of the additional information. Their research showed that integrating several latent features into a tense classifier could improve the performance of the tense classifier, while the tense classifier using only latent features also outperformed that using surface features. Toma and Saddiq [8] designed a model that took both source and target tense information into consideration. They proposed a temporal model under classification technology, to deal with the issue of temporal translation consistency that there were no obvious tense markers in some source language, but the temporal information in the target language was easy to get. Kasper et al. [9] pointed out that MT based on artificial intelligence fundamentally changed the public's understanding and attitude towards multilingual communication. In some language pairs, the accuracy, quality, and efficiency of some types of machines translated text may be quite high. Therefore, the acceptability of users and their dependence on MT content are reasonable. However, if MT is used in a high-risk environment without understanding its shortcomings, key evaluations, and modifications to the original output, MT in small and/or low resource languages may produce significantly low quality, which may lead to potential negative consequences and risks [10–13].

Through literature review, it can be found that although the processing of tense in Chinese-English MT has achieved some results, it is basically carried out on a small-scale corpus. It is difficult to obtain large-scale labeled data with these methods. Therefore, a Chinese-English temporal annotation algorithm based on deep learning is put forward, which extracts the temporal information of Chinese phrases based on deep belief network.

## 2. Methods

### 2.1. Chinese Verb Tense Recognition Based on Long Short-Term Memory (LSTM)

#### 2.1.1. Related Researches about Chinese Temporal Annotation

The automatic annotation of Chinese tenses is a common issue in Chinese language processing. With the rise of MT, researchers have begun to pay attention to the transformation and transmission of Chinese and English tenses. The problem lies in the recognition of Chinese tenses, and there have been many related studies.

Kim and Won [14] constructed all verbs in a Chinese sentence into a verb vector according to their positions in the sentence. Each verb in the vector was attached with relevant semantic and grammatical features, and then the determination of the tense of each verb in the Chinese sentence was transformed into the serialized annotation. They first constructed a small-scale human-annotated dataset containing tense transformations from Chinese linguistic data to English linguistic data. Then a temporal classifier on the ground of linear conditional random field was trained for temporal annotation of the Chinese linguistic data. Their method covered complex linguistic phenomena through statistical machine learning and considered the annotation of tense of each verb as a whole. Finally, an accuracy of 58.21% was reported for the temporal annotation.

Riloff and Jones [15] come up with a Chinese verbal tense recognition method based on a self-training algorithm. They obtained English verbal tenses from the English part-of-speech tagging and then converted the English tenses of the parallel corpus into Chinese verbal tenses through word alignment information, to form the original training dataset. Then, the dataset was used to train a support vector machine (SVM) classifier, and the self-training algorithm was applied to filter the data and strengthen the model. In the final experimental results they reported, the accuracy of temporal classification reached 77.49%.

Although the above methods have achieved good results in Chinese temporal annotation, the original training data they used were basically completed by manual annotation, so it was difficult to reproduce their work. Moreover, the experiments were carried out on small-scale corpora, and it was also difficult to obtain large-scale labeled data with these methods. Therefore, in the data preparation of this research, another new method is adopted to obtain a large number of Chinese corpora with temporal information. The Attention soft alignment information of the traditional neural MT model is utilized, and the corresponding Chinese tense is obtained from the part-of-speech tagging results of the English corpus.

#### 2.1.2. Chinese Temporal Annotation Based on LSTM

As the main in-depth learning framework in the process of processing neurolinguistic programming (NLP), LSTM makes up for the deficiency of cyclic NN and can effectively solve the gradient disappearance problem, and the special hidden unit contained therein can effectively preserve the long-term information of text, which is very suitable for processing text objects with time series characteristics [16, 17]. Compared with traditional machine learning, LSTM has better processing efficiency for Chinese text and can intuitively express the essential characteristics of language. Chinese text sentences contain temporal information. When using LSTM model to obtain text information, it will also obtain the temporal information contained in text verbs. Therefore, for the tense prediction of Chinese verbs, LSTM model has a good processing effect [18]. The sixteen tenses of English verbs are shown in Table 1.

The LSTM prediction model mainly includes softmax layer, full connection layer, dropout layer, LSTM layer, and embedding layer. Its basic composition is illustrated in Figure 1.

Each Chinese word in the sentence is converted to network input through the embedding layer, and then the output of the LSTM network is processed through the softmax layer and the full connection layer, and finally the temporal prediction information of the current word is obtained. The operation process of the whole model is to receive the input of a Chinese word sequence and then generate the temporal classification sequence of the corresponding position.

Dropout method is adopted to prevent overfitting during data training. Dropout method is not training for a single network, but training the whole deep neural network and averaging the results of the whole set. The probability of abandoning some neurons by deep neural network is *p*, while the probability of remaining other neurons is *q* = 1 − *p*, and the output of abandoned neurons is set to 0.

#### 2.1.3. Model Enhancement Algorithm Using Bootstrapping

Because the original training data is relatively rough, the annotation results of Chinese tense contain a lot of noise. In order to strengthen the training model and improve the model effect, bootstrapping algorithm is used to reduce the impact of noise data. Bootstrapping algorithm is a uniform sampling algorithm. Specifically, after selecting a sample in the training set, the sample may be added to the training set again [19].

The bootstrapping algorithm is simplified. Because a large amount of labeled data is needed in the process of NN training, the initial data set is too large, rather than a small amount of manual labeled data in traditional machine learning. Some data in the training set is not completely random extraction, but by gradually expanding the number of samples in the training set and then cleaning the training data; by adding the sample to the training set through iterative learning process, some restrictions such as “removing sentences without verbs” are set.

#### 2.1.4. Neural Machine Translation (NMT) Model Combined with Automatic Temporal Classification of Source Verbs

The trained Chinese verb temporal classification model is applied to the translation process of NMT. The temporal classification results of Chinese verbs and the English verb tenses generated by translation are defined as Ta and Tb, respectively. In order to obtain the tense of the target English word, the part of speech of the target word table needs to be marked first, and then each word in the word table is obtained through the Chinese and English word tense acquisition algorithm. Finally, a tense table corresponding to the word sequence number in the word table is formed [20]. Encoder-Decoder model framework is given in Figure 2.

In the Decoder stage, if the source position corresponding to the current time step is a verb, the constraint *T*_*a*_=*T*_*b*_ is added to the beam-search process. The model structure is shown in Figure 3.

*a*, *b*, *c*, *d*, *e*, *f*, and *g* represent the Chinese text input at the source side to be translated, the output results of the Chinese temporal annotation model, the Encoder and Attention structures in the simplified NMT system, the Decoder network of NMT, the output of the Decoder network at the target side, the list of words to be selected in the beam-search search process, and the final generated translation. Through the process shown in Figure 3, the temporal information of the source side is transmitted to the target side through the Attention structure, and the temporal categories of verbs generated in each step are guided, so that the translation tenses of the source side and the target side are consistent.

#### 2.1.5. Experiment Setting

Opennmt, the open-source framework for neural MT, is used to train the baseline model, and the model translation results are improved through the Chinese temporal annotation results. During the training process, any new information is not introduced, and the neural machine is trained to translate 13 epochs according to the steps given in the official instructions of Opennmt. The main parameters and descriptions used to train the baseline model are shown in Table 2.

The training process of the baseline model is simply to train a NMT system containing advanced modules. In this process, no temporal information is added, and the temporal information of Chinese verbs at the source is not involved in the training process. Before the translation of the test set, it first annotated the Chinese of the test corpus in advance through the Chinese temporal annotation model and only extracted the temporal sequence of the corresponding sentences in the translation process.

### 2.2. Deletion and Recovery of Tense

In the task of natural language processing, the order of words is crucial, and the change of order may lead to the change of the meaning of the whole sentence. Position coding is usually trained according to specific tasks, and in the Transformer model, position coding is calculated by

(1) $$\begin{array}{c} {\text{PE}}_{\left(\text{pos},2i\right)}=\sin\left(\frac{\text{pos}}{10000^{2i/d_{\text{model}}}}\right),\\ {\text{PE}}_{\left(\text{pos},2i+1\right)}=\cos\left(\frac{\text{pos}}{10000^{2i/d_{\text{model}}}}\right). \end{array}$$

#### 2.2.1. Detemporal Algorithm

Detemporal algorithm is to remove the tenses of verbs in English sentences, convert them into simple present tenses, and give them real singular and plural forms. It is often used in the construction of tenseless translation systems. The mutual transformation between the original English corpus and the nontemporal English corpus can be completed by the detemporal algorithm [21].

Because the form of Chinese verbs is stable, when tense changes, the form of Chinese verbs will not change, so it does not do tense processing on Chinese corpus. Moreover, since the words corresponding to time adverbs and auxiliary words in Chinese sentences cannot be found in the timeless English sentences in the training process, the model will automatically ignore the temporal information in Chinese sentences [22].

Dependency relations in English sentences can be obtained by dependency syntax tree or phrase syntax analysis tree [23, 24]. Taking “iron tree, worker, learning, English, grammar” as an example, the dependency syntax tree and phrase analysis syntax tree are illustrated in Figure 4.

After getting the dependency relationship in the sentence, it can be detemporalized by “marking-arranging.” Marking process is to locate and judge the verb tense through the dependency relationship in the sentence, find out the words related to the verb tense, and mark them. Marking is divided into temporal transformation marking and deletion marking. The deletion marking is represented by TENDEL, indicating that the corresponding words need to be deleted. The temporal transformation marking indicates that the tense of the corresponding words needs to be transformed into the simple present tense. If the part of speech of the word is different, the corresponding marking is also different.

The arranging process refers to the processing of words marked in the marking process and deleting words related to tense in the sentence, such as the copula in present continuous tense and “have” in present perfect tense, which need to be deleted, and the words that need to be transformed are transformed into simple present tense and corresponding singular or plural form.

#### 2.2.2. Temporal Recovery Algorithm

In order to map the temporal information of the Chinese translation to the corresponding English verbs and obtain the English sentences with final tense, after getting marked Chinese tense tree, Chinese-English alignment relation, and tenseless English sentences, tense recovery is needed. Alignment relation is an array. By combining Chinese and English sentence sequences and traversing alignment relation array, English verbs and corresponding Chinese words are obtained [25]. Then, it traverses the Chinese syntax analysis tree from the bottom up to find the node where the Chinese words correspond to the English verbs and then finds the temporal information of the corresponding clause node or the corresponding node in the Chinese tense tree. If the Chinese word corresponding to the English verb is a verb, the English verb is transformed to make its form correspond to the tense of the Chinese verb. If the Chinese word corresponding to English verb is not verb, then when transforming English verb, it is necessary to make its morphology correspond to the tense of the clause in which Chinese word is located. When transforming the form of English verbs, it is necessary to judge whether the English verbs will be affected by other words. For example, when there are copulas, modal verbs, and connectors before the verbs, the form of English verbs will not be treated [26]. The algorithm flowchart is shown in Figure 5.

#### 2.2.3. Chinese-English Alignment

Chinese-English alignment is the bridge between tenseless English sentences and Chinese tense tree, and it is also the key of Chinese-English tense translation system. The accuracy of the process will directly affect the accuracy of the translation results. English verbs in tenseless English sentences can find the corresponding pretranslation Chinese verbs through Chinese-English alignment and then obtain the tense of the verb through the Chinese tense tree.

The Chinese-English alignment relation needed in the Chinese-English tense translation system is a two-dimensional matrix, while what is obtained through the Chinese-English tenseless translation system is a four-dimensional matrix. Therefore, the two-dimensional alignment matrix is obtained after processing the four-dimensional matrix by the feature superposition method. Firstly, after the integration of six eight-head alignment matrices, six two-dimensional matrices are obtained. Then, after fusing six two-dimensional matrices, a two-dimensional matrix fusing 48 alignment matrices is obtained. Finally, the obtained two-dimensional matrix is numerically binarized, and the matrix is traversed column by column. The maximum value in a column is set to 1, and the other values are set to 0.

Taking into account the needs of the subsequent temporal recovery algorithm, the obtained binary alignment matrix is transformed into an alignment array consistent with the length of English sentences. Each number in the array corresponds to the position of words in Chinese sentences. In order to get the alignment array, it is necessary to annotate the part of speech in English sentences. Through the annotation results, the alignment information of English words as verbs in the alignment matrix is retained, and the subscript value of the Chinese word corresponding to the English verb is added to the number and stored in the position corresponding to the English verb in the array. For the corresponding English words in the array, the positions of nonverbs are set to zero, indicating that English words on these positions are not involved in the recovery process.

#### 2.2.4. Data Preprocessing

Transformer model needs to train both DeTense and baseline models. Baseline model data preprocessing is included in DeTense model preprocessing. Therefore, it mainly introduces the preprocessing process of DeTense model. The main steps of the preprocessing process are given in Figure 6:

- Step 1: label removal: because the data is labeled data, the corresponding rules are needed to extract the required content.
- Step 2: word segmentation: this process is the primary task in the process of MT. Chinese and English data need to be processed and are segmented by Jieba and Mose.
- Step 3: symbol processing: the brackets in Chinese and English data are processed, and all English brackets are changed into Chinese brackets, so as to avoid the syntactic analysis errors caused by brackets.
- Step 4: syntactic analysis: in order to generate the data of de-emporal operation, Berkeley parser is needed for the syntactic analysis of English data.
- Step 5: DeTense: English syntax analysis tree is entered in the DeTense program, and the English word segmentation sentences before and after the DeTense are obtained after processing. The format is ANSI. After the process is finished, the text editing tool is used to convert the encoding format to UTF8.
- Step 6: screening: the detemporalized English word segmentation sentences are traversed to find the ROOT in the sentences. The corresponding Chinese and English sentences before and after DeTense are deleted according to the location information of ROOT.

#### 2.2.5. Experiment Setting

The performance of tense translation system in Chinese-English translation task is studied. The experimental training data adopted 4.16 million Chinese-English parallel sentence pairs in the second edition of the Chinese-English parallel corpus of the United Nations. Validation and test data were selected from 3,434 Chinese-English parallel sentence pairs provided by the official website of the United Nations Corpus. The above data are label data, which need to be processed by preprocessing.

Transformer model is used to construct NMT system. After processing the data through different processing methods, two corpora of temporal and nontemporal are obtained. Data with tense are used to train the baseline model, and data without tense are used to train the DeTense model. Combined with the Chinese-English temporal annotation algorithm, the translation with tense can be obtained.

BLEU is used to evaluate the translation results and multi-bleu.per1 script is used to calculate. The parameter settings of the experimental network are as follows: model=transformer; vocab − size=32*K*; batch − size=1024; beam − size=4; alpha=0.6; train − steps=500*K*.

## 3. Results and Discussion

### 3.1. NMT Experiment Combined with Temporal Annotation

Through the statistics of the original training data, the statistics of Chinese temporal annotation results are shown in Figure 7.

A model under Chinese tense classification is added to the neural MT process, and the results obtained are shown in Table 3.

The translation results can be effectively improved by adding the Chinese tense recognition at the source to the NMT model, and the translation effect of the neural machine model will also be affected by the results of Chinese verb tense recognition to a certain extent. The average results of the standard LSTM Chinese temporal annotation model are basically consistent with the baseline, but the general trend remains unchanged, and both are rising. However, in the NIST04 test set, the test results of all models are not ideal, which may be affected by model adaptability.

The bidirectional LSTM Chinese temporal annotation model is more accurate in predicting Chinese verb tenses, and the improvement effect of NMT model is also obvious. Good test results are obtained in all test sets. For the temporal annotation task of Chinese verbs, the accuracy of the double-layer LSTM model is similar to that of the standard LSTM model, and the improvement effect on the NMT model is also limited. Compared with the results of the tagging LSTM model on the test set, there are also fluctuations, and the overall prediction results are not much different.

### 3.2. Comparison of Model Translation Effect

In this section, the temporal annotation algorithm is added to the translation process of the timeless translation system trained by the Transformer model. The final translation effect is compared with the baseline translation system. The results are given in Figure 8.

As the current mainstream translation model, the multiheaded attention mechanism in Transformer model can focus on some temporal information and better deal with Chinese-English tense translation. Whether in the test set or the verification set, there is still a certain gap between the model test effect and the baseline effect.

The correct example sentences of the experiment are shown in Table 4.

The example sentences in Table 4 describe the state at a certain moment in the future, so the verb “减少” in the original Chinese sentence should be of the simple future tense. The tense tagging algorithm obtains tense-related features from the original Chinese sentence and determines that the tense of the verb “will be reduced” is of simple future tense by constructing a probability model of the entire tense tree corresponding to the original Chinese sentence. Thus, “is reduced” in the tenseless English sentence is changed to “will be reduced,” and the correct translation is obtained; while the baseline model fails to obtain the sentence tense accurately and the translation is biased. It should be noted that the values in the table are not filled in errors, but are caused by the translation not processing the values. Examples of translation errors are shown in Table 5.

Table 5 displays an example of a translation error, from which it can be found that the method proposed in this research obtains the simple future tense actually. But the translation of verbal tense is biased due to the error of Chinese-English alignment.

## 4. Conclusions

With the rapid development of computer technology and modern linguistics, MT research has made new progress, and many commercial and practical MT systems have emerged. Tense translation is a very important task in MT. Due to the different information entropy between Chinese and English, the current Chinese-English MT system is not much effective. This is mainly due to the difficulty in understanding Chinese sentences, so the difficulty in transforming Chinese sentences into English sentences is relatively high. In short, the development of deep learning has made a breakthrough in the development of MT, but tense is still an urgent problem to be solved in MT, especially in Chinese-English MT.

A Chinese verb temporal annotation model is proposed. Firstly, in order to obtain Chinese verb tense, the NN is used to construct the Chinese temporal annotation model. In the process of translation, the source tense is passed to the target through the alignment matrix of the traditional Attention mechanism, and the probability of translation candidates in the candidate translation set that are inconsistent with the corresponding source text tense is reduced. Then, the Chinese-English temporal annotation algorithm is integrated into the MT model to construct a Chinese-English translation system with temporal processing function. The essence of this system is to use the Chinese-English temporal annotation algorithm to obtain the temporal information from Chinese sentences and transmit it to the corresponding English sentences in the translation process, to realize the tense processing of English sentences and obtain the English sentences corresponding to the original Chinese sentences.

However, the current work is at the sentence level, and in the temporal processing, discourse information also plays a vital role. For example, the beginning of an article is “in 2005,” so the whole article needs to use the past tense. The research on the combination of discourse information is not yet mature, and more people will participate in this work in the future.

## Figures and Tables

**Figure 1:** Automatic Chinese temporal annotation model based on LSTM.

**Figure 2:** Encoder-Decoder model framework.

**Figure 3:** NMT model.

**Figure 4:** Structure diagram (a) dependency syntax tree; (b) phrase analysis syntax tree.

**Figure 5:** Flow chart of temporal recovery algorithm.

**Figure 6:** DeTense model data preprocessing steps.

**Figure 7:** Chinese temporal annotation results.

**Figure 8:** Comparison of model translation effect (a) translation effect of the last model; (b) average translation effect of the last 10 models.

**Table 1:** Sixteen tenses of English verbs.

Tense	Simple tense	Perfect tense	Continuous tense	Perfect continuous tense
Present tense	Simple present tense	Present perfect tense	Present continuous tense	Present perfect continuous tense
Past tense	Simple past tense	Past perfect tense	Past continuous tense	Past perfect continuous tense
Future tense	Simple future tense	Future perfect tense	Future continuous tense	Future perfect continuous tense
Past future tense	Simple past future tense	Past future perfect tense	Past future continuous tense	Past future perfect continuous tense

**Table 2:** Main parameter settings and descriptions of baseline model training.

Parameters	Parameter value	Descriptions
Scr vocab size	30000	The size of source Chinese vocabulary
Tgt vocab size	30000	The size of target English vocabulary
Batch size	64	Minibatch size, the number of training samples taken out for each training
Embedding size	500	Dimensions of source and target word embedding
Encoder type	BiLSTM	The type of neural network used by Encoder, a bidirectional LSTM here
Decoder type	LSTM	The neural network type used by Decoder, the standard LSTM used here
Enc/Dec layers	2	Network layers of Encoder and Decoder
LSTM size	500	Dimension of hidden layer of the neural network in LSTM
Optimization	Adam	Type of the optimization functions
Learning rate	0.001	Learning rate for neural network training
Beam size	10	The size of each candidate set selected in beam-search

**Table 3:** Test results of NMT model combined with source-side Chinese annotation information.

Models	NIST03	NIST04	NIST05	NIST06	NIST08	Mean value
Baseline	35.84	38.84	34.46	33.85	26.59	33.92
Tense-LSTM	35.76	38.40	34.56	34.59	26.74	34.01
Tense-BiLSTM	35.99	38.67	34.70	34.92	26.76	34.21
Tense-2layers	36.06	38.56	34.43	34.52	26.85	34.08

**Table 4:** Correct experimental example sentences.

Original Chinese sentence	因此, 经常预算准备金总数将减少至3.484亿美元
Original English sentence	Thus, total regular budget reserves will be reduced to $348.4 million
Baseline	The total reserve for the regular budget would be reduced to $348.4 million
Tenseless English sentence	The total level of the regular budget reserve is reduced to $484.4 million
DeTense + temporal annotation	The total level of the regular budget reserve will be reduced to $484.4 million

**Table 5:** Examples of experimental errors.

Original Chinese sentence	即便如此, 如果这将使我们能够更好地了解历史问题及其法律内涵, 再次把不满化为友谊, 那么, 用同情和宽容看待各种讨论, 并期待各方抱有同样的态度, 也是理所当然的。
Original English sentence	Even so, if this will enable us to better understand historical issues with their legal aspects and to transform resentment into friendship again, it is natural to approach different discourses with empathy and tolerance and expect a similar attitude from all sides
Baseline	Even so, if this will enable us to better understand the historical issues and their legal dimensions, to turn the grievances once again into friendship, then it is legitimate to view the discussion with compassion and tolerance and to expect the same attitude from all sides
Tenseless English sentence	Even so, if it enables us to better understand historical issues and their legal content and once again translate grievances into friendship, then it is only natural to view the discussions with sympathy and tolerance and to expect the same attitude on all sides
DeTense + temporal annotation	Even so, if it enables us to better understand historical issues and their legal content and once again will translate grievances into friendship, then it is only natural to view the discussions with sympathy and tolerance and to expect the same attitude on all sides

## Data Availability

The data used to support the findings of this study are included within the article.
